# Effects of Enalapril on TLR2/NF-*κ*B Signaling Pathway and Inflammatory Factors in Rabbits with Chronic Heart Failure

**DOI:** 10.1155/2021/9594607

**Published:** 2021-07-13

**Authors:** Yanping Tang, Zelin Xu, Xinyu Chen, Nan Wang, Xu Deng, Liqi Peng, Qingyang Chen, Huzhi Cai

**Affiliations:** ^1^Hunan University of Chinese Medicine, Changsha, Hunan 410208, China; ^2^The First Hospital of Hunan University of Chinese Medicine, Changsha, Hunan 410007, China

## Abstract

Chronic heart failure (CHF) refers to the state of persistent heart failure, which is a complex clinical syndrome of various advanced heart diseases. The toll-like receptor 2 (TLR2)/nuclear transcription factor-*κ*B (NF-*κ*B) signal transduction pathway is one of the pathological mechanisms of CHF. Adriamycin can significantly induce the upregulation of TLR2 expression. Angiotensin-converting enzyme inhibitors (ACEI) are commonly used drugs for the treatment of CHF. In our study, the CHF model was established by injection of doxorubicin into the rabbit ear vein. The effect of enalapril on the TLR2/NF-*κ*B signaling pathway in CHF rabbits has been analyzed and determined. Our research results showed that enalapril reduced the inflammatory response by inhibiting the activation of the TLR2/NF-*κ*B signaling pathway, thereby improving cardiac structure, myocardial remodeling, and cardiac function.

## 1. Introduction

Chronic heart failure (CHF) is a complex clinical syndrome in the end stage of various heart diseases. It is the ultimate fate and main cause of death for most cardiovascular diseases. CHF usually deteriorates rapidly; the prognosis is poor; and the mortality rate is high, which five-year survival rate is similar to that of malignant tumors. Studies have shown that immune-inflammatory response and inflammatory cell infiltration are one of the pathological mechanisms of CHF. The inflammatory response is an essential factor in promoting myocardial remodeling and cardiac function deterioration, which can be an independent predictor of disease progression and prognosis. The toll-like receptor 2 (TLR2)/nuclear transcription factor-*κ*B (NF-*κ*B) signaling pathway is an important pathway in the body's inflammatory system. It is widely found in various tissues and cells and is involved in the occurrence and regulation of various diseases. Recent studies have found that adriamycin can significantly induce the upregulation of TLR2 expression when replicating heart failure models, resulting in excessive activation of TLR2 downstream signaling pathways such as NF-*κ*B [1]. Activated NF-*κ*B can also promote myocardial remodeling under certain conditions. Moreover, the heart can express a variety of inflammatory cytokines during CHF, and the NF-*κ*B pathway is one of the mechanisms for activation, production, and sustained release of inflammatory cytokines [2]. Angiotensin-converting enzyme inhibitors (ACEI) are commonly used drugs for the treatment of CHF. Previous studies have shown that ACEI can inhibit angiotensin-converting enzyme (ACE), reduce the production of angiotensin II (Ang II), inhibit the excessive activation of neuroendocrine, improve ventricular remodeling, reduce cardiac load, and improve cardiac function. However, its mechanism needs further study. In this study, we established the CHF rabbit model by injecting adriamycin into the ear vein. We observed the effect of enalapril on the TLR2/NF-*κ*B signaling pathway in CHF rabbits through molecular biological technology to explore further the protective effect of enalapril on chronic heart failure and its mechanism.

## 2. Materials and Methods

### 2.1. Animals

Male New Zealand rabbits, weighing 1.7∼2.0 kg, were purchased from the experimental animal center of the Hunan University of Chinese Medicine (animal license number: SCXK (Xiang) 2009∼0012). Each rabbit was fed for one week under the conditions of free diet, light/dark cycle of 12 h/12 h (light time of 6:00∼18:00), the background noise of 40 ± 10 dB, and environment temperature of 20 ± 3°C.

### 2.2. Experimental Methods

#### 2.2.1. Preparation of a Chronic Heart Failure Model

Adriamycin hydrochloride for injection was diluted into a solution of 1 mg/mL with normal saline and injected into the ear vein of the rabbit at a concentration of 1 mL/kg each time. According to the rabbit's weight, the dose of doxorubicin was adjusted twice a week for 8 weeks [3]. At the end of the fourth week, cardiac function was measured by color Doppler ultrasound to determine whether the CHF model was established successfully.

#### 2.2.2. Grouping and Administration

Among the 35 New Zealand rabbits, 11 were randomly selected as the normal control group. The remaining 24 rabbits were treated with intravenous adriamycin to replicate the CHF model according to the above modeling method. At the end of the fourth week, the surviving New Zealand rabbits were stratified according to cardiac function and then randomly divided into the model group and the enalapril group. The enalapril group was given enalapril 5 mg/kg by gavage (according to the conversion of human and rabbit body surface area) starting from the fifth week [4]. The normal control group and the model group were given the same amount of distilled water by gavage every day. It lasted four weeks.

#### 2.2.3. Echocardiographic Examination

The same ultrasound technician performed all tests. The rabbits were anesthetized by intravenous injection of 25% urethane at a dose of 4 ml/kg. The ultrasound probe was placed on the left sternal border and the long axis of the left ventricle to obtain the maximum diameter. Portable software automatically calculated left ventricular ejection fraction (LVEF), left fractional ventricular shortening (LVFS), the ratio of peak E to peak A (E/A), left ventricular end-diastolic diameter (LVDD), left ventricular end-systolic diameter (LVSD), interventricular septal thickness (IVS), and left ventricular posterior wall thickness (LVPW). And the study reported an average of 5 heartbeat cycles.

#### 2.2.4. Measurement of Myocardial Hypertrophy Index, Heart Weight Index, (HWI) and Left Ventricular Weight Index (LVWI)

After anesthesia, the rabbit's body weight (BW) was weighed by an electronic balance, and its heart was quickly removed by thoracotomy, and its heart weight (HW) was weighed. The great vessels, the left and right atria, and the right and left ventricles were separated along the atrioventricular junction. The filter paper absorbed the water; the left ventricular weight (LVW) was measured; and the myocardial hypertrophy index was calculated. HWI = HW/BW and LVWI = LVW/BW.

#### 2.2.5. Extraction of Total Protein from Myocardial Tissue

The 100 mg left ventricular myocardial tissue was cut into small pieces and placed into a centrifuge tube. The tissue lysate was added into the centrifuge tube in a ratio of about 1:8 (mass: volume). The centrifuge tube was placed in the ice bath, mechanically homogenized, eddy mixed, stood for 1 h, centrifuged at 18,000 g, and kept at 4°C for 30 min, and the supernatant was taken to be the total protein of the tissue. The protein concentration of lysates was classified by the Bradford method, then packaged separately, and stored at −80°C for later use.

#### 2.2.6. Western Blotting

50 *μ*g of total myocardial proteins were added to 2x SDS sample buffer (0.1 mol/L Tris, pH 6.8, 0.2 mol/L DTT, 4% SDS, 20% glycerol, and 0.02% bromophenol blue). The mixture was denatured at 100°C for 8 min, and then the sample was loaded. Electrophoresis was carried out at 16 mA/gel for the first 15 minutes and then to the bottom at 32 mA/gel. The current was set to 0.8 mA/cm^2^ for electroblotting according to the membrane area. The protein was transferred to the nitrocellulose membrane for 2 hours. Then, the nitrocellulose membrane was blocked with TBST containing 3% nonfat dry milk for 2 hours at room temperature. The membrane was removed and placed in a hybridization bag. Anti-TLR2 and anti-NF-*κ*B antibodies were added separately. The bag was stored at 4°C overnight. After rinsing was performed three times with TBST (10 minutes each), the membrane was removed and placed in another hybridization bag. The enzyme-labeled secondary antibody was added, and the hybridization was carried out at room temperature for 2 hours. Rinsing was performed three times with TBST (10 minutes each). The membrane was exposed to the chemiluminescent solution, imaged, and scanned at 300 dpi. The ratio of the gray value of TLR2 and NF-*κ*B protein to the gray value of GAPDH protein indicated the relative expression level of TLR2 and NF-*κ*B protein.

#### 2.2.7. Detection of Serum Indexes

Blood samples were collected from the middle ear artery in every group. After standing for 10 minutes, the blood was centrifuged at 3,000 rpm for 15 minutes, and the serum was separated and stored in a refrigerator at –80°C. The concentrations of N-terminal pro-B-type natriuretic peptide (NT-proBNP), tumor necrosis factor-*α* (TNF-*α*), and matrix metalloprotein-9 (MMP-9) were determined by ELISA kits according to the manufacturer's instructions.

#### 2.2.8. Statistical Method

The statistical software SPSS 19.0 was used for statistical analysis. The measurement data were all expressed by “mean ± standard deviation” ($\bar{x}\pm s$). The comparison between multisample means was tested by one-way ANOVA. The *t*-test was used for comparison between two groups. *P* < 0.05 indicates that the difference is statistically significant.

## 3. Results

### 3.1. Changes in the Number of Experimental Rabbits

Among the total of thirty-five New Zealand rabbits, two rabbits died of excessive anesthesia in the first four weeks. Before the end of the experiment, one rabbit in the model group and one in the enalapril group died of diarrhea.

### 3.2. Effects of Enalapril on Left Ventricular Function Indexes of Rabbits

LVEF, LVFS, and E/A in the model group were significantly decreased than those in the normal control group (*P* < 0.05). Compared with the model group, LVEF, LVFS, and E/A in the enalapril group were significantly increased (*P* < 0.05), indicating that enalapril can significantly improve the heart function of CHF rabbits as shown in Figure 1.

### 3.3. Effect of Enalapril on Morphological Indexes of the Left Ventricle in Rabbits

Compared with the normal control group, LVDD, LVSD, IVS, and LVPW in the model group were significantly increased (*P* < 0.05 and *P* < 0.01). Compared with the model group, LVDD, LVSD, IVS, and LVPW were decreased significantly in the enalapril group (*P* < 0.05 and *P* < 0.01) as shown in Figure 2.

### 3.4. Effects of Enalapril on HWI and LVWI in Rabbits

Compared with the normal control group, HWI and LVWI in the model group were significantly increased (*P* < 0.05 and *P* < 0.01). Compared with the model group, both HWI and LVWI in the enalapril group were significantly reduced (*P* < 0.01), suggesting that enalapril can significantly reverse myocardial hypertrophy of the rabbits with CHF as shown in Figure 3.

### 3.5. Effect of Enalapril on the Expression of TLR2 and NF-*κ*B Protein in Rabbit Myocardium

Compared with the normal control group, the expression of TLR2 and NF-*κ*B protein in the model group was significantly increased (*P* < 0.01). Compared with the model group, the expression of TLR2 and NF-*κ*B protein in the enalapril group was decreased (*P* < 0.05) as shown in Figures 4 and 5.

### 3.6. Effect of Enalapril on the Serum NT-proBNP, TNF-*α*, and MMP-9 in Rabbits

Compared with the normal control group, the levels of serum NT-proBNP, TNF-*α*, and MMP-9 in the model group were significantly increased (*P* < 0.05 and *P* < 0.01). Enalapril can significantly reduce the levels of serum NT-proBNP, TNF-*α*, and MMP-9 (*P* < 0.05 and *P* < 0.01) as shown in Figure 6.

## 4. Discussion

Ventricular remodeling is the main pathological feature of CHF and also an important reason for the deterioration of cardiac function in patients with CHF. The immune inflammatory response plays a key role in the process of ventricular remodeling and tissue fibrosis. The toll-like receptor (TLR) is a new type of pattern recognition receptor. It is a bridge connecting innate immunity and adaptive immunity and participates in the body's innate immune response. The signaling pathway induced by TLRs plays an important role in ventricular remodeling. TLRs expression is most widely expressed in more than 20 kinds of cells, mainly expressed in skeletal muscle and myocardium. After TLRs receptors are activated, TLR2 mainly participates in the occurrence and development of atherosclerosis by promoting the inflammatory reaction, extracellular matrix (ECM) degradation, and intimal hyperplasia [5, 6]. The knockout of the TLR2 gene has no significant effect on the infarct area and the degree of inflammatory cell infiltration in the infarct area. Still, it can reduce myocardial fibrosis and ventricular remodeling in the noninfarct area [7]. Inhibition of TLR2 can improve adriamycin-induced cardiac dysfunction by regulating inflammatory response and apoptosis pathway [1]. Therefore, TLR2 may be an effective intervention target in the treatment of heart failure. After TLR2 is activated, the signal is transmitted through Mal and MyD88, and finally, NF-*κ*B is activated, thereby promoting the expression of inflammatory cytokines.

NF-*κ*B is a dimeric protein that is widely existed in eukaryotes. As the hub of signal pathways, it is closely related to the regulation of immunity, tumors, apoptosis, and embryonic development. It is an important nuclear transcription factor and plays an important mediating role in the inflammatory reaction [8]. The activation of NF-*κ*B plays an essential role in the pathogenesis of CHF. It can specifically bind to the enhancer *κ*B sequence of the immunoglobulin *κ* light chain gene to regulate the expression of a series of inflammatory factors [9]. The overexpression of NF-*κ*B can activate BNP, TNF-*α*, and MMP-9; affect the degradation balance of the extracellular matrix; and promote cardiomyocyte hypertrophy, ventricular remodeling, cardiac cavity enlargement, and CHF [10, 11].

NT-proBNP is a peptide hormone composed of 76 amino acids, which can be dissociated from the precursor of BNP. When the ventricular wall tension or pressure increases, the secretion of NT-proBNP increases. It mainly reflects the changes in ventricular pressure and volume load and is closely related to the severity of heart failure. NT-proBNP is an important evaluation index for the diagnosis, severity, and prognosis of CHF [12]. TNF-*α* is an inflammatory factor secreted mainly by mononuclear macrophages and also an important transmitter of the body's immune response and inflammatory response. In chronic heart failure, the heart is both TNF-*α* synthesis and the target organ for its action. In the process of chronic ventricular remodeling after myocardial infarction, cardiomyocytes will produce large amounts of TNF-*α*. TNF-*α* can further activate the NF-*κ*B-induced enzyme and promote NF-*κ*B to enter the nucleus, thereby activating the expression of a series of genes required for cell inflammation, growth, and survival [13]. Matrix metalloproteinases (MMPs) are a family of enzymes that can specifically degrade ECM components and are the main factors causing tissue collagen remodeling. MMP-9 is one of the key enzymes in the degradation of the myocardial extracellular matrix and is closely related to ventricular remodeling [14, 15]. Studies have shown that NF-*κ*B activation can increase the expression of MMP-9, cause ECM deposition, and promote the formation of glomerular fibrosis [16].

In this study, the CHF model was replicated by injecting adriamycin into the ear vein. Compared with the normal control group, LVEF, LVFS, and E/A of the rabbits in the model group were significantly decreased, and LVDD, LVSD, IVS, LVPW, HWI, and LVWI were significantly increased, and the levels of NT-proBNP, TNF-*α*, and MMP-9 were significantly increased. These results suggest that the chronic heart failure model was successfully reproduced. Western blot results showed that the expression levels of TLR2 and NF-*κ*B protein in the rabbit myocardium in the model group were significantly higher than those in the normal control group, indicating that ventricular remodeling and cardiac dysfunction of CHF are related to the overexpression of TLR2 and NF-*κ*B proteins. It was found that LVEF, LVFS, and E/A were significantly increased. While LVDD, LVSD, IVS, LVPW, HWI, and LVWI were significantly reduced, NT-proBNP, TNF-*α*, and MMP-9 levels were also decreased significantly. The results of this study showed that enalapril could significantly ameliorate the ventricular remodeling and cardiac function of CHF rabbits and reduce the level of inflammatory factors. Western blot results showed that the expression of NF-*κ*B and TLR2 protein in the myocardial tissue of the enalapril group was significantly downregulated. TLR2 can recognize pathogens in innate immunity and trigger the body's immune response to pathogenic microorganisms, thereby generating cascade reactions. After a series of reactions, NF-*κ*B nuclear displacement occurred, and NF-*κ*B could upregulate the expression of NT-proBNP, TNF-*α*, MMP-9, and other inflammatory factors. Lee et al. [17] showed that enalapril could inhibit NF-*κ*B in intestinal epithelial cells and peritoneal macrophages of mice and alleviate experimental colitis. The research by Kim et al. also showed that enalapril inhibited NF-*κ*B-induced inflammation in aged rats [18]. The results of this study showed that enalapril could reduce the expression of TLR2 and NF-*κ*B protein; reduce the level of inflammatory factors such as NT-proBNP, TNF-*α*, and MMP-9, and inhibit the inflammatory response of CHF rabbits, thereby delaying the abnormal remodeling of the myocardial interstitium and ultimately protecting the cardiac function, which are consistent with partial research results of Lee and Kim et al. [17, 18].

## 5. Conclusion

In summary, during chronic heart failure, the expression of TLR2 and NF-*κ*B protein in myocardial tissue was significantly enhanced; the levels of inflammatory factors such as NT-proBNP, TNF-*α*, and MMP-9 were significantly increased; and ventricular remodeling and cardiac diastolic and systolic dysfunction occurred. Enalapril significantly inhibited ventricular remodeling, improved cardiac function, inhibited the secretion of inflammatory factors, and downregulated the expression of TLR2 and NF-*κ*B protein. The results of this study suggested that enalapril reduced inflammation by inhibiting the activation of the TLR2/NF-*κ*B signaling pathway, thereby improving cardiac structure, myocardial remodeling, and cardiac function. This might be the potential biological mechanism of enalapril in the treatment of CHF, which needed further study in the future.

## Figures and Tables

**Figure 1:** Changes of left ventricular function indexes of rabbits in every group after the experiment. Note: compared with the normal control group, ^*∗*^*P* < 0.05; compared with the model group, ^Δ^*P* < 0.05.

**Figure 2:** Changes of left ventricular morphological indexes of rabbits in every group after the experiment. Note: compared with the normal control group, ^∗^*P* < 0.01 and ^∗∗^*P* < 0.01; compared with the model group, ^Δ^*P* < 0.05 and ^ΔΔ^*P* < 0.01.

**Figure 3:** Effects of Enalapril on HWI and LVWI in rabbits. Note: Compared with the normal control group, ^∗^*P* < 0.01 and ^∗∗^*P* < 0.01; compared with the model group, ^ΔΔ^*P* < 0.01.

**Figure 4:** Expression of TLR2 and NF-*κ*B protein (gray value ratio) in myocardium of rabbits in every group after the experiment. Note: compared with the normal control group, ^∗∗^*P* < 0.01; compared with the model group, ^Δ^*P* < 0.05.

**Figure 5:** Electrophoretogram of NF-*κ*B and TLR2 protein expression in myocardium of rabbits in every group.

**Figure 6:** Changes of serum NT-proBNP, TNF-*α* and MMP-9 levels in rabbits of every group after the experiment. Note: compared with the normal control group, ^∗^*P* < 0.05 and ^∗∗^*P* < 0.01; compared with the model group, ^Δ^*P* < 0.05 and ^ΔΔ^*P* < 0.01.

## Data Availability

The data sets used and/or analyzed during the current study are available from the corresponding author on reasonable request.
